# DL-MRI: A Unified Framework of Deep Learning-Based MRI Super Resolution

**DOI:** 10.1155/2021/5594649

**Published:** 2021-04-09

**Authors:** Huanyu Liu, Jiaqi Liu, Junbao Li, Jeng-Shyang Pan, Xiaqiong Yu

**Affiliations:** ^1^School of Electronics and Information Engineering, Harbin Institute of Technology, Harbin 150001, China; ^2^Center of AI Perception, AI Research Institute, Harbin Institute of Technology, Harbin 150001, China; ^3^College of Computer Science and Engineering, Shandong University of Science and Technology, Qingdao 266590, China; ^4^32021 Troops of the PLA, Beijing 100094, China

## Abstract

Magnetic resonance imaging (MRI) is widely used in the detection and diagnosis of diseases. High-resolution MR images will help doctors to locate lesions and diagnose diseases. However, the acquisition of high-resolution MR images requires high magnetic field intensity and long scanning time, which will bring discomfort to patients and easily introduce motion artifacts, resulting in image quality degradation. Therefore, the resolution of hardware imaging has reached its limit. Based on this situation, a unified framework based on deep learning super resolution is proposed to transfer state-of-the-art deep learning methods of natural images to MRI super resolution. Compared with the traditional image super-resolution method, the deep learning super-resolution method has stronger feature extraction and characterization ability, can learn prior knowledge from a large number of sample data, and has a more stable and excellent image reconstruction effect. We propose a unified framework of deep learning -based MRI super resolution, which has five current deep learning methods with the best super-resolution effect. In addition, a high-low resolution MR image dataset with the scales of ×2, ×3, and ×4 was constructed, covering 4 parts of the skull, knee, breast, and head and neck. Experimental results show that the proposed unified framework of deep learning super resolution has a better reconstruction effect on the data than traditional methods and provides a standard dataset and experimental benchmark for the application of deep learning super resolution in MR images.

## 1. Introduction

MRI [1] is a type of tomography, which uses magnetic resonance to obtain electromagnetic signals from the human organ tissue and reconstruct human information about the structure of human organs. MRI has been used in imaging diagnosis of various systems throughout the body, including craniocerebral [2], spinal cord [3], large heart blood vessels [4], joint bones [5], and soft tissues and pelvis [6]. High-resolution MR images have richer structural details, which is helpful for doctors to locate the lesions and diagnose the disease. The acquisition of MR high-resolution image needs to increase the magnetic field intensity and pulse radiation time, high intensity magnetic field, and ultra-long pulse radiation not only bring bad experience to patients but also produce image artifacts due to patients' movement, thus affecting the quality of imaging. Therefore, the software method for MR image super resolution has great significance, and it can improve the MR image resolution without causing harm to the human body.

Super resolution is to restore high-frequency detail from low-resolution image to improve image resolution. The simplest method is to use interpolation to improve the image resolution, such as bicubic interpolation [7] and nearest neighbor interpolation [8]. However, the interpolation method is not in essence to increase the image information, so it cannot recover the image high-frequency information. Subsequently, people put forward the super-resolution method based on spatial domain constraints because this algorithm has wide applicability and strong prior constraint capability. In this respect, algorithms include reverse iterative projection method [9–11], statistical method based on maximum posterior probability [12–14], nonuniform sample interpolation method [15, 16], and convex set projection method [17]. These algorithms make full use of spatial correlation of data, introduce fuzzy, point diffusion, and other degradation parameters into image degradation model, and cover global motion and local motion. However, when dealing with the super resolution of multiframe images, the quality of reconstructed images declines rapidly as the super-resolution ratio increases or the number of available input images decreases. Under such circumstances, the reconstructed results will appear too smooth and lack important high-frequency details.

The learn-based super-resolution method is different from the image priori knowledge acquired under various assumptions. It directly learns the image priori knowledge from a large number of samples. The learning-based image super-resolution methods mainly include dictionary learning [18] and deep learning [19]. In dictionary learning, a high-resolution image block can utilize a high-resolution dictionary sparse representation, and the sparse coefficient can be obtained from the sparse representation of the low-resolution dictionary of the corresponding low-resolution image block. However, the super-resolution method based on sparse representation needs to solve the sparse representation of the super-complete dictionary. When the dictionary size or reconstructed image size is large, the computational time complexity is still very high, which still has a considerable gap with the real-time application. The super-resolution method based on deep learning has been validated in natural images. The network used by NISR mainly includes three categories: feedforward deep networks, feedback deep networks, and generative adversarial networks. DBPN [20] belongs to the feedforward deep network, which provides an error feedback and interdependent modules, which represent image degradation and high-resolution, making characteristics of the sampling phase are connected to improve the SR result. RDN [21] belongs to the feedback deep network. It proposes a residual dense block (RDB) and uses the densely connected convolutional layer to extract rich local features. SRFBN [22] belongs to the feedback deep network. This type of model implements this feedback method by using hidden states in constrained RNNs. EDSR [23] also belongs to the feedback deep network. Compared with SRResNet in structure, EDSR removes the batch normalization (BN) operation. SRGAN [24] is a generative adversarial network. It takes the residual network as the main network of feature extraction and adds the perceptive loss function. Alternate training generates network and discriminant network. The three major types of representative networks have made good contributions to super-resolution reconstruction of natural images.

At present, some deep learning methods are also applied to MR image super resolution. Chen et al. [25] apply DenseNet to brain MRI image super resolution, Chen et al. [26] propose a novel 3D CNN architecture, namely, mDCSRN, which provides appealing sharp SR images with rich texture details that are highly comparable with the referenced HR images.

We compared and analyzed bicubic, RDN, EDSR, SRGAN, DBPN, and SRFBN, algorithms on the constructed MR image dataset, covering traditional super-resolution learning and a batch of deep learning networks with excellent super-resolution performance. As can be seen from the experimental results, the super-resolution effect of the deep learning network on the MR image performs well, and the super-resolution effect of different parts of the same algorithm fluctuates greatly.

Our contributions include the following three points:

1. We proposed a unified framework of deep learning-based MRI super resolution and carried out an experimental analysis of the traditional super-resolution methods and deep learning super-resolution methods on the MRI dataset.
2. We build a dataset for super resolution of MR images, including 4300 high-low resolution pairs. It involves the skull, breasts, knees, and head and neck.
3. We performed statistical analysis on the difficulty of MR images in different parts and provided suggestions for MR images in different parts.

## 2. A Unified Framework of Deep Learning and Dataset

### 2.1. Image Degradation

Because of tissue and organ movement in the process of imaging, the existence of the noise and artifacts makes image or part of the image blur, or resolution is not enough, so by the imaging model [27, 28], the low-resolution image is the high-resolution image by ideal after deformation, fuzzy, blood sampling, such as noise adding income after operation, and process of image degradation process.  Figure 1 shows the degradation process of high-resolution images. *X* is an undergraded high-resolution image matrix with an ideal band limit not lower than Nyquist sampling frequency. Let *x* be the column vector of *X*. After the degradation process of *x*, such as deformation matrix *M*_*k*_, fuzzy matrix *B*_*k*_, and mass reduction sampling matrix *D*_*k*_, noise matrix *n*_*k*_ is added to obtain the low-resolution image *y*_*k*_. The mathematical model formula of image degradation is shown in Figure 1:

(1) $$\begin{array}{c} y_{k}=D_{k}B_{k}M_{k}x+n_{k},\;1\leq k\leq p. \end{array}$$

Formula (1) can also be expressed as

(2) $$\begin{array}{c} Y=HX, \end{array}$$

where *H* represents the image degradation matrix, *Y* represents low-resolution images, and *X* represents ground truth high-resolution images. The purpose of image super resolution is to find the inverse of the degenerate matrix *H*.

### 2.2. A Unified Framework of Deep Learning-Based MRI Super Resolution

We propose a unified framework of deep learning-based MRI super resolution. The aim of this framework is to apply the deep learning network for natural image super resolution to MR images. We have integrated five state-of-the-art deep learning networks, respectively, Deep Backprojection Networks For Super Resolution (DBPN), Residual Dense Network (RDN), Feedback Network for Image Super Resolution (SRFBN), Photo-Realistic Single Image Super-Resolution Using a Generative Adversarial Network (SRGAN), and Enhanced Deep Residual Networks for Single Image Super Resolution (EDSR). The unified framework of deep learning-based MRI super resolution is shown in Figure 2.

DBPN: the structure of DBPN is shown in Figure 2(a). It consists of initial feature extraction, projection, and reconstruction.conv(*f*, *n*) represents the convolution layer, *n* represents the number of filters, and *f* represents the filter size.

Initial feature extraction: we use 3^*∗*^3 convolution to extract features from low-resolution images. Then, we use 1^*∗*^1 convolution to achieve feature reduction. *n*_0_ is the number of filters used in the initial LR feature extraction phase. *n*_*R*_ is the number of filters used in each projection unit.

Backprojection stages: from Figure 2(A), the main component of the DBPN structure is the projection unit. As part of training the SR system, it maps LR features to HR features, or maps HR features to LR features in two opposite mapping relationships. The two mapping relationships are

(3) $$\begin{array}{c} \text{Upsampling: }H_{0}^{t}=\left(L^{t-1}*p_{t}\right)↑s, \end{array}$$

(4) $$\begin{array}{c} \text{Downsampling: }L_{0}^{t}=\left(H^{t-1}*g_{t}\right)↓s, \end{array}$$

(5) $$\begin{array}{c} \text{Residual: }e_{t}^{l}=L_{0}^{t}-L^{t-1}, \end{array}$$

(6) $$\begin{array}{c} \text{Residualup sampling: }H_{1}^{t}=\left(e_{t}^{l}*q_{t}\right)↑s, \end{array}$$

(7) $$\begin{array}{c} \text{Output feature map: }H^{t}=H_{0}^{t}+H_{1}^{t}. \end{array}$$

The above formula ^*∗*^ represents a convolution operation, ↑*s* stands for up sampling operation, ↓*s* stands for down sampling operation, and *p*_*t*_, *g*_*t*_, *q*_*t*_ is the (de) convolutional layer of the stage *t*, which learns the mapping of low-resolution feature maps to high-resolution feature maps.

Reconstruction: the feature diagrams obtained by each reflection unit are connected to form [*H*^1^, *H*^2^,…, *H*^*t*^]. And, the combined features are transformed into reconstructed images by 3∗3 convolution.

RDN: it can be seen from (B) Figure 2 that RDN network is composed of SFENet, RDBs, DFF, and UPNet. SFENet is composed of two convolutional layers for extracting shallow features. RDBs module is composed of the residual block and the dense block. This operation facilitates the training of RDB modules with larger growth rates. DFF module consists of global feature fusion and global residual learning, which realizes the global extraction of the characteristics of each layer. UPNet implements image upsampling.

SRFBN: we can see from (C) in Figure 2 that the network is mainly an improvement of a feedback mechanism based on the DRCN large framework, which is equivalent to turning the weight-sharing layer in DRCN into a weight-sharing module and add a skip connection. It consists of three parts: feature extraction, weight-sharing module, and learning strategy.

1. Feature extraction: this network is mainly for shallow feature extraction, that is, shallow feature extraction is *F*_in_^*t*^=*f*_LRFB_.
2. Weight-sharing module: the output of the *t* weight-sharing module should be *F*_out_^*t*^=*f*_*FB*_(*F*_out_^*t*−1^, *F*_in_^*t*^), and the corresponding intermediate supervision output is *I*_SR_^*t*^=*I*_Res_^*t*−1^+*f*_UP_(LR), among them, *I*_Re*s*_^*t*^=*f*_RB_(*F*_out_^*t*^).
3. Learning strategy: the learning supervision function used by this model is as follows:

(8) $$\begin{array}{c} L\left(\Theta \right)=\frac{1}{T}{\sum_{t=1}^{T}W^{t}\left\|I_{HR}^{t}-I_{SR}^{t}\right\|}_{1}. \end{array}$$

The truth value of the intermediate supervision will be selected according to the difficulty of the task, such as a single bicubic downsampling degradation, and all truth values are the same; for BD (bicubic + blur) degradation, the first two intermediate supervised outputs use truth values with Gaussian blur, and the subsequent intermediate supervises use truth values without Gaussian blur.

SRGAN: it can be seen from Figure 2(D) that SRGAN is composed of the generator, discriminator, and loss function.

The generator is composed of multiple residual blocks in the generated network part (SRResNet). Each residual block is composed of two 3 × 3 convolution layers, the batch normalization layer (BN), PReLU as the activation functions are the latter items of the convolution layer, and two subpixel convolution layers.

The discriminator consists of 8 convolutional layers in the discriminating network part, and LeakyReLU is selected as the activation function. The role of the discriminator is to determine the difference between the high-resolution image output by the generator and the real high-resolution image.

The loss function in SRGAN is more special than other networks. It uses two loss functions: *G* loss and *D* loss. *G* loss and *D* loss can be expressed as

(9) $$\begin{array}{c} l^{\text{SR}}=l_{X}^{\text{SR}}+10^{-3}l_{\text{Gen}}^{\text{SR}}, \end{array}$$

(10) $$\begin{array}{c} \underset{\theta_{G}}{\min}\underset{\theta_{D}}{\max}E_{I^{\text{HR}}∼p_{\text{train}}\left(I^{\text{HR}}\right)}\left[\log\;D_{\theta_{D}}\left(I^{\text{HR}}\right)\right]+E_{I^{\text{LR}}∼p_{G}\left(I^{\text{LR}}\right)}\left[\log\left(1-G_{\theta_{G}}\left(I^{\text{LR}}\right)\right)\right]. \end{array}$$

It can be seen from the above formula that *l*_*X*_^*SR*^ is content loss and 10^−3^*l*_*Gen*_^*SR*^ is against loss. The losses of the two are

(11) $$\begin{array}{c} l_{\text{MSE}}^{\text{SR}}=\frac{1}{r^{2}WH}\sum_{x=1}^{rW}\sum_{y=1}^{rH}{\left(I_{x,y}^{\text{HR}}-G_{\theta_{G}}{\left(I^{\text{LR}}\right)}_{x,y}\right)}^{2}, \end{array}$$

(12) $$\begin{array}{c} l_{\text{VGG}/i,j}^{\text{SR}}=\frac{1}{W_{i,j}H_{i,j}}\sum_{x=1}^{W_{i,j}}\sum_{y=1}^{H_{i,j}}{\left(\phi_{i,j}{\left(I^{\text{HR}}\right)}_{x,y}-\phi_{i,j}G_{\theta_{G}}{\left(I^{\text{LR}}\right)}_{x,y}\right)}^{2}. \end{array}$$

EDSR: it can be seen from (E) in Figure 2 that it is similar to SRResnet, but the structure lacks a ReLU layer and a batchnorm layer, mainly, because the batch normalization layer normalizes the function. Therefore, by normalizing the functions, the scope flexibility of the network can be eliminated. Because the structure adopted by this method is too deep, the instability of the training process can easily cause numerical instability. To solve this problem, the model uses residual scaling to deal with it, by which the last convolutional layer output of the residual module is multiplied by 0.1.

### 2.3. Dataset for Training

We collected the MR image data of the four body parts of the head and neck, breast, bones, and skull on the open source website and used the bicubic downsampling method to construct high-low resolution MR image pairs of different scales, including ×2, ×3, and ×4, and divided the training set, validation set, and test set according to 7 : 2 : 1.

#### 2.3.1. Collection and Quality Filtering of Raw Datasets

Our data comes from open source MR image data, including NYU fastMRI Dataset [29], IXI Dataset [30], TCIA MRI Dataset [31], and mridata.org [32]. Because different datasets include different parts, some data contain only one human body part. For example, NYU fastMRI dataset contains the skull and knee, IXI dataset contains the skull only, and TCIA MRI dataset contains the breast, skull, head and neck, and bladder. Therefore, this dataset is mainly based on the MRI image data downloaded from TCIA. The skull data also comes from NYU fastMRI dataset and IXI dataset; the knee parts are from mridata.org and NYU fastMRI dataset.

MR image data is stored in DICOM format, which is an international standard for medical images. We used *Python*'s third-party library pydicom to parse the obtained raw MR data. Thus, MR images of various organs are acquired. The MR image information of each part is shown in Table 1.

To reduce the impact caused by the signal-to-noise ratio, contrast, motion artifacts, and chemical artifacts of the image and in addition to considering the cost borne by the MRI equipment, we collect and use the mainstream magnetic field strength. Because we acquire data of different parts, according to different imaging standards of medical target organs, we obtain original images with different resolutions.

As shown in Table 1, we obtained a large amount of raw MR image data, but not all data are suitable for MR image super resolution. Unqualified data will reduce the effect of image super resolution. Therefore, we conducted a quality assessment of the data obtained for each organ and proposed data that did not meet the requirements. We screened MR images using both manual and machine methods.

Firstly, according to the advice of professional doctors, we manually removed the MR image data with obvious quality problems. Secondly, the performance of deep learning algorithm is positively correlated with the quality and quantity of data. However, more samples do not mean better performance. Poor quality data will not help the deep learning training, but will reduce the quality of reconstructed images. In this paper, we used a method based on gray consistency and gradient combined to evaluate MR image quality. The number of filtered images is shown in Table 1. The filtered data will be used as the training data of deep learning.

#### 2.3.2. Training Set Generation

Various types of deep learning networks need to be based on prior knowledge which is a pair of high-low resolution MR images. We adopt the downsampling method based on the bicubic method. Downsampling based on cubic interpolation first requires the construction of a bicubic function. Its expression is

(13) $$\begin{array}{c} W\left(x\right)=\left\{\begin{array}{cc} \left(a+2\right){\left|x\right|}^{3}-\left(a+3\right){\left|x\right|}^{2}+1, & \text{for}\left|x\right|\leq 1,\\ \left(a+2\right){\left|x\right|}^{3}-5a{\left|x\right|}^{2}+8a\left|x\right|-4a, & \text{for}1<\left|x\right|<2\text{,}\\ \text{0,} & \text{otherwise.} \end{array}\right. \end{array}$$

Secondly, to treat the interpolated image points, take the nearby 4 × 4 area. Interpolate as follows.

(14) $$\begin{array}{c} f\left(x,y\right)=\sum_{i=0}^{3}\sum_{j=0}^{3}f\left(x_{i},y_{j}\right)W\left(x-x_{i}\right)W\left(y-y_{j}\right). \end{array}$$

Thirdly, the image obtained by upsampling is processed by downsampling, and the corresponding downsampling is

(15) $$\begin{array}{c} g\left(x,y\right)=f\left(x,y\right)↓, \end{array}$$

The HR is the original image. *g*(*x*, *y*) is the LR image obtained by downsampling.

In order to simulate the real MR image acquisition process, we sampled HR images down and added Gaussian noise to obtain corresponding LR images. The downsampling method based on LR plus noise is to add the original image without noise and add 5% Gaussian noise to the LR image obtained after downsampling:

(16) $$\begin{array}{c} \text{HR}↓s⟶{\text{LR}}_{s}+5\%\text{GN}. \end{array}$$

Among them, 5%GN represents 5% of Gaussian noise. LR_*s*_+5%GN represents low-resolution images of *s* size corresponding to this method.

We use the method of direct downsampling of the original image based on cubic interpolation to generate MR-SR high-low resolution pairs as input to the deep learning network. We mainly use the bicubic downsampling to implement the HR- > LR process. The downsampling scales of the dataset are ×2, ×3, and ×4. The generated multiscale MR image training set is shown in Figure 3.

## 3. Experimental Results and Analysis

### 3.1. Experimental Setup and Evaluation Index

#### 3.1.1. Experimental Setup

During the training process, the hardware configuration we used is Core i9-9900K processor and dual-pass 1080ti graphics card, 32G memory. The software configuration is super-resolution network training using pytorch framework. We set the parameters of the 5 types of networks and iterate 200 rounds. Set the learning rate to 0.01, and its network parameter setting table is shown in Table 2. We found that the learning rates of the five models were fine-tuned within a certain range, and they all reached convergence before 200 rounds of training iterations. After 200 rounds of training, the losses of the five models hardly changed. For better comparative analysis, we set the same number of iterations.

#### 3.1.2. Evaluation Index

In this paper, PSNR and SSIM are used to comprehensively measure the effect of MR image super-resolution reconstruction.

PSNR: this evaluation standard is the most commonly used. The higher the PSNR, the better the reconstructed image quality. The calculation formula is as follows:

(17) $$\begin{array}{c} \text{MSE}=\frac{1}{MN}{\left\|X-Y\right\|}^{2}, \end{array}$$

where *X* stands for the high-resolution image, *Y* represents the reconstructed image, *M* and *N*, respectively, represent the height and width of the image, and *L* represents the largest gray value in the gray level, where *L*=255.

SSIM: this evaluation indicates the degree of structural similarity between the reconstructed image and the original image. The larger the value, the more similar the reconstructed image and the original image and the better the reconstruction effect. The calculation formula is

(18) $$\begin{array}{c} \text{SSIM}\left(X,Y\right)={\left[l\left(X,Y\right)\right]}^{\alpha }{\left[c\left(X,Y\right)\right]}^{\beta }{\left[s\left(X,Y\right)\right]}^{\gamma }, \end{array}$$

where *l*(*X*, *Y*) stands for the brightness contrast operator, *c*(*X*, *Y*) stands for the contrast operator, *s*(*X*, *Y*)stands for the structure contrast operator, and *α*, *β*, *γ* > 0 is used to adjust the weights of the three operators. The calculation formulas are as follows.

Brightness contrast operator:

(19) $$\begin{array}{c} l\left(X,Y\right)=\frac{2\mu_{x}\mu_{y}+C_{1}}{\mu_{x}^{2}+\mu_{y}^{2}+C_{1}},\\ C_{1}={\left(K_{1}L\right)}^{2}. \end{array}$$

Contrast operator:

(20) $$\begin{array}{c} c\left(X,Y\right)=\frac{2\sigma_{x}\sigma_{y}+C_{2}}{\sigma_{x}^{2}+\sigma_{y}^{2}+C_{2}},\\ C_{2}={\left(K_{2}L\right)}^{2}. \end{array}$$

Structure contrast operator:

(21) $$\begin{array}{c} s\left(X,Y\right)=\frac{\sigma_{xy}+C_{3}}{\sigma_{x}\sigma_{y}+C_{3}},\\ C_{3}={\left(K_{3}L\right)}^{2}, \end{array}$$

where *μ* represents the average value of the image, that is, the average brightness of the image, *σ* represents the standard deviation of the signal and estimates the contrast of the signal, *C* represents the normalization factor that overcomes zero, and *K* is a constant. The mean *μ* and variance *σ* are calculated as

(22) $$\begin{array}{c} \mu_{x}=\frac{1}{MN}\sum_{i=1}^{MN}x_{i}, \end{array}$$

(23) $$\begin{array}{c} \sigma_{x}=\sqrt{\frac{1}{MN}\sum_{i=1}^{MN}{\left(x_{i}-\mu_{x}\right)}^{2}}. \end{array}$$

### 3.2. Experimental Result and Analysis

After training of various deep network models, the results obtained by each model in our MR dataset have obvious manifestations. As can be seen from Figure 4 and Table 3, the SRGAN algorithm is richer in visual texture. The SRFBN algorithm is better at the PSNR and SSIM indicators. We can draw this conclusion. First of all, for the same network, the SR effect of different organ parts is significantly different, which is mainly caused by the original resolution of each organ, the magnetic field intensity during the acquisition process, and the proportion of free water and bound water in the organ. Secondly, we can customize a network specifically adapted to this organ for different parts. For example, in Table 3, although the RDN network does not perform well in the head and neck, breast, knee, and other organs, this network obviously has a better PSNR/SSIM of 38.05/0.9565 in the skull organs than other networks, indicating that different target organs can be customized to design super-resolution networks.

We can see from the table that the PSNR/SSIM index between the traditional bicubic algorithm and the deep network is particularly different, which is basically between 3.61–12.59/0.1896–0.2951, which also shows that the deep network has better image super-resolution reconstruction effect on MR image super resolution. It can be seen through experiments that directly applying deep learning networks can also achieve certain effects, indicating that deep networks have a certain role in MR image super resolution and are better than traditional methods. However, there is still a gap with the super-resolution effect of natural images. The main reason is that the natural image and MR image have different imaging mechanisms. Therefore, it is necessary to combine the characteristics of MR images of different human parts to design a more targeted deep super-resolution network of MR images.

We made statistics on the number of parameters and calculation amount of the five deep learning methods, as shown in Table 4.

It can be seen from Table 4 that the model parameters and calculation amount of different networks differ greatly. Combined with the super-resolution performance of the five methods in Table 3, the SRFBN method not only has better super resolution effect but also has the least model size and calculation amount, which is more suitable for practical application.

## 4. Conclusion

We propose a unified framework of deep learning-based MRI super resolution. We have integrated five state-of-the-art deep learning networks. Moreover, the deep learning method is experimentally verified on the self-built MR image dataset which covers the skull, knee, breast, and head and neck. Through data quality screening and analog imaging degradation, MR image dataset with certain scale and standard for image super resolution is formed. Compared with the traditional method, the deep learning method has better reconstruction performance on the data set. The reason of the difference of the super resolution of different organs is revealed from the structure level of each organ. We hope that our paper can provide data support for the application of deep learning networks in MR super resolution and inspire future research on MR image super resolution.

## Figures and Tables

**Figure 1:** Image degradation model.

**Figure 2:** A unified framework of deep learning-based MRI super resolution.

**Figure 3:** MR image super-resolution pairs, including three different high-low resolution pairs of MR images.

**Figure 4:** HR comparison of different super-resolution deep networks for each MRI data with scale = 4.

**Table 1:** Sorting of raw MR data.

Data name	Magnetic field strength (T)	Resolution	Raw/filtered data
Knee	1.5	256^*∗*^256	4517/1000
Skull	3.0	256^*∗*^256	7917/2200
Breast	1.5	288^*∗*^288	3816/600
Head and neck	3.0	512^*∗*^512	2653/500

**Table 2:** Parameter settings of each network.

Parameter	RDN	EDSR	GAN	FBN	DBPN
Lr	0.0001	0.0001	0.0001	0.0001	0.0001
bath_size	64	64	128	64	128
Number of iterations	200	200	200	200	200
Activation	Relu	Relu	Leak	Relu	Relu
	Relu				

**Table 3:** PSNR/SSIM of MRI dataset on different networks.

Dataset	Scale	Bicubic	RDN	EDSR	SRGAN	D-DBPN	SRFBN
Head and neck	×2	25.44/0.6928	29.05/0.8824	37.34/0.9861	37.69/0.9868	35.74/0.9800	38.03/0.9879
	×3	23.04/0.6289	27.41/0.8326	31.14/0.8693	—/—	31.61/0.9474	32.79/0.9595
	×4	21.58/0.5442	24.53/0.7144	29.25/0.9164	28.78/0.9093	29.28/0.9182	30.23/0.9304

Breast	×2	28.56/0.8848	33.50/0.9373	34.57/0.9447	34.06/0.9332	31.94/0.9243	34.28/0.9428
	×3	21.85/0.6130	30.61/0.8876	31.25/0.8949	—/—	28.56.0.8568	32.14/0.9040
	×4	20.50/0.4830	23.68/0.6118	30.00/0.8631	27.99/0.8137	28.13/0.8351	30.68/0.8735

Knee	×2	30.60/0.9185	36.34/0.9641	37.49/0.9719	36.93/0.9670	37.67/0.9727	37.95/0.9744
	×3	24.36/0.6202	32.13/0.9103	32.85/0.9230	—/—	33.75/0.9360	33.82/0.9377
	×4	22.69/0.5649	30.02/0.8597	28.34/0.8968	29.63/0.8643	31.29/0.8940	31.35/0.8964

Skull	×2	20.320.6025	38.05/0.9565	38.03/0.9565	35.80/0.9234	33.82/0.9062	39.19/0.9600
	×3	19.23/0.5843	28.81/0.7790	34.16/0.9211	—/—	31.38/0.8620	35.65/0.9300
	×4	18.60/0.5623	29.70/0.7962	32.22/0.8886	30.95/0.8500	29.39/0.7906	33.60/0.9089

**Table 4:** Model parameter estimation and calculation capabilities.

Methods	RDN	EDSR	SRGAN	D-DBPN	SRFBN
Param (M)	22.317	43.103	214.376	10.426	3.546
FLOPs (T)	7.43	11.71	15.32	4.27	0.94

## Data Availability

The two popular MRI datasets in this paper, fastMRI Dataset and IXI Dataset can be freely downloaded from https://fastmri.org/and http://www.brain-development.org/.
